RETRACTED

# Artificial Intelligence-Based Feature Analysis of Ultrasound Images of Liver Fibrosis

**DOI:** 10.1155/2022/2859987

**Published:** 2022-07-30

**Authors:** Youcheng Xie, Shun Chen, Dong Jia, Bin Li, Ying Zheng, Xiaohui Yu

**Affiliations:** ^1^Department of Gastroenterology, The 940 Hospital of Joint Logistic Support Force of PLA, Lanzhou 730050, China; ^2^The First Clinical Medical School, Gansu University of Chinese Medicine, Lanzhou 730000, China

## Abstract

Liver fibrosis is a common liver disease that seriously endangers human health. Liver biopsy is the gold standard for diagnosing liver fibrosis, but its clinical use is limited due to its invasive nature. Ultrasound image examination is a widely used liver fibrosis examination method. Clinicians can diagnose the severity of liver fibrosis according to their own experience by observing the roughness of the texture of the ultrasound image, and this method is highly subjective. Under the premise that artificial intelligence technology is widely used in medical image analysis, this paper uses convolutional neural network analysis to extract the characteristics of ultrasound images of liver fibrosis and then classify the degree of liver fibrosis. Using neural network for image classification can avoid the subjectivity of manual classification and improve the accuracy of judging the degree of liver fibrosis, so as to complete the prevention and treatment of liver fibrosis. Therefore, the following work is done in this paper: (1) the research background, research significance, research status at home and abroad, and the impact of the development of medical imaging on the diagnosis of liver fibrosis are introduced; (2) the related technologies of deep learning and deep convolutional network are introduced, and the indicators of liver fibrosis degree assessment are constructed by using ultrasonic image extraction features; (3) using the collected liver fibrosis dataset to conduct model evaluation experiments, four classic CNN models are selected to compare and analyze the recognition rate. The experiments show that the GoogLeNet model has the best classification and recognition effect.

## 1. Introduction

Liver disease is a major clinical problem, and the ability to accurately diagnose it is critical in the treatment of patients. For example, there are two types of liver diseases: localized lesions and diffuse lesions. In focal liver disease, the lesions are concentrated in a small area of liver tissue, while in diffuse lesions, the lesions are located throughout the liver. The most common kind of liver disease, with major consequences for public health, is called diffuse liver disease [1]. Liver fibrosis is the most common type of diffuse liver disease, which refers to the pathological process of liver connective tissue hyperplasia caused by chronic diseases or other reasons and eventually liver cirrhosis [2]. Liver fibrosis is reversible. If liver fibrosis is detected and treated in time, it can still return to normal. Otherwise, it will be difficult to cure once it develops into liver cirrhosis [3]. The quantitative staging system for liver fibrosis can not only diagnose whether there is liver fibrosis in time and reduce the risk of liver fibrosis patients transforming into cirrhosis but also provide a certain reference for doctors to observe the effect of drug treatment and facilitate doctors to adjust the dose of drugs; it has important clinical significance. According to the Chinese Medical Association's guidelines for the prevention and treatment of viral hepatitis, fibrosis can be divided into five stages: *S*0, *S*1, *S*2, *S*3, and *S*4. Among them, *S*0 represents no liver fibrosis, *S*4 represents liver cirrhosis, and *S*1–*S*3 in the middle represent different degrees of liver tissue lesions [4]. Liver biopsy is the gold standard for clinical diagnosis of the severity of liver fibrosis, but biopsy is a traumatic examination that causes not only pain but also bleeding, and many patients are reluctant to undergo biopsy. Moreover, it may cause misdiagnosis due to sampling error and these shortcomings limit its application in the diagnosis of liver fibrosis [5]. Ultrasound image examination has the characteristics of noninvasiveness, convenience, high repeatability, no radiation, and low price and is one of the widely used liver examination methods [6]. After fibrosis occurs in some tissue parts of the liver, the absorption and reflection properties of ultrasound in these tissue parts will also change. The ultrasound signal reflected by the liver tissue is converted by the ultrasound diagnostic apparatus, and the resulting ultrasound image of the liver will also change. These changes mainly include roughening of the liver parenchyma, thickening of the hepatic vein wall, and sharpening of the liver capsule margin [7]. In the ultrasound images of normal rat livers and liver ultrasound images of cirrhotic rats, it can be seen that the liver parenchyma becomes rough. However, other changes, such as thickening of the hepatic vein wall and sharpening of the capsular margin, are not evident in the picture. This is because in the actual ultrasound examination process, due to the limitations of equipment and the proficiency of the operating doctor, the characteristics of some fibrotic lesions, such as the hepatic vein wall and the edge of the capsule, are difficult to reflect in the ultrasound image. Therefore, clinicians mainly make the diagnosis of fibrosis based on the roughness of liver ultrasound images. Doctors can diagnose the severity of liver fibrosis based on their own experience by observing the thickness of the echoes in the ultrasound images, combined with the shear wave velocity value [8]. This method is highly subjective and can only diagnose hepatic fibrosis qualitatively. Not only can it not subdivide the 5 stages of fibrosis, it is also insensitive to the effect of drug treatment, and it may cause misdiagnosis and delay the treatment of patients. There is a clinical need for an automatic diagnosis system that can extract the characteristics of the echo thickness of the liver from ultrasound images and perform quantitative staging of fibrosis. Moreover, it is required that the quantitative staging of fibrosis is as fine as possible, and it is better to divide 5 stages more accurately, which can not only improve the diagnostic accuracy of fibrosis but also has great significance for the observation of drug treatment effects. Under the premise that artificial intelligence technology is widely used in medical image analysis, this paper uses the convolutional neural network analysis to extract the characteristics of ultrasound images of liver fibrosis and then classify the degree of liver fibrosis. Using neural network for image classification can avoid the subjectivity of manual classification and improve the accuracy of judging the degree of liver fibrosis, so as to complete the prevention and treatment of liver fibrosis. Therefore, the work done in this paper has great practical significance.

RETRACTED

## 2. Related Work

Clinically, the main role of various auxiliary examinations is to perform fibrosis staging for chronic liver disease to determine whether there is liver fibrosis and its severity. After the diagnosis of liver fibrosis or even liver cirrhosis, clinicians will initiate screening and monitoring procedures and formulate a comprehensive treatment plan [9]. These methods can also follow up patients who have been diagnosed with fibrosis, predict whether patients with liver cirrhosis will develop significant portal hypertension, and can also be used to evaluate the efficacy of patients after antiviral and liver fibrosis treatment, providing evidence for the formulation of clinical treatment plans [10]. Ultrasound is currently one of the most commonly used examination techniques for evaluating chronic liver disease [11]. The advantages are that it is noninvasive, objective, reproducible, real-time, simple, and inexpensive and is not affected by the metal machinery placed in the patient, which has been widely accepted. Ultrasound can now provide information on liver morphology and hemodynamics as well as tissue physical properties such as liver stiffness or elastic modulus, making it one of the most important noninvasive methods for evaluating liver fibrosis in recent years with the extensive development of new technologies such as ultrasound elastography and contrast-enhanced ultrasound [12]. There are three main methods for noninvasive assessment of liver fibrosis by ultrasound elasticity: transient elastography (TE), real-time tissue elastography imaging (RTE), and point quantification and two-dimensional shear wave elastography (pSWE and 2DSWE). Acoustic radiation force impulse (ARFI) is applied in both pSWE and 2DSWE [13]. All technicians performing elastic ultrasound operations need to go through a relevant learning curve, master the corresponding basic knowledge, have experience in conventional ultrasound operations, and undergo specialized elastic ultrasound training. During the examination, the patient needs to hold his breath. Holding his breath in a resting state is the guarantee for obtaining the best measurement value. Deep inhalation, Valsalva breathing, and deep exhalation will all change the hepatic venous pressure and affect the elasticity value of liver stiffness [14]. TE is a technology that indirectly measures the liver stiffness value by measuring the propagation velocity of the shear wave excited by the vibration of the patient's skin by a low-frequency mechanical source, thereby reflecting the degree of liver fibrosis. Vibration-controlled transient elastography (VCTE) produced by FibroScan company in the United States is currently the most commonly used assessment method for liver fibrosis [15]. In addition, VCTE has been validated in large-scale clinical trials of various liver diseases, and it is recommended to use VCTE in hepatitis B patients rather than serological indicators for liver fibrosis assessment [16]. RTE is to apply an internal or external dynamic or static pressure to the tissue. Under the action of elasticity, biomechanics, and other factors, the displacement of the tissue before and after the compression will change. By calculating the change of this displacement and using ultrasonic imaging methods and digital image processing techniques, tissue stiffness can be estimated using strain elastography [17]. HITACHI has developed a piece of software for quantitative analysis of tissue diffusion, selects ROI in the elastic image, and divides the color in the region into 256 levels. The horizontal and vertical coordinates represent the number of color levels and frequency distribution of strain values, respectively. Strain histograms were used to evaluate 11 parameters of the liver based on the amount of fibrotic features extracted from image texture features, and then the liver fibrosis index (LFI) was analysed according to these 11 parameters, which is used to reflect the degree of liver fibrosis. RTE can avoid the intrahepatic large vascular structure, and it is its advantage to select the liver parenchyma for imaging and quantitative detection. Moreover, obese patients and patients with ascites can be imaged, which has certain clinical application prospects [18]. SWE includes point quantification pSWE and 2DSWE. Using acoustic radiation pulses to generate transverse shear waves at different depths in the body, the propagation speed of shear waves in different soft tissues is different, so by measuring the propagation speed, the elastic value of tissue hardness can be directly calculated, and the color carrying the information can also be the codes which are superimposed on 2D anatomical images, allowing qualitative and quantitative detection of regions of interest [19]. In addition to the above ultrasound methods for evaluating liver fibrosis, CT perfusion imaging is also a new method to indirectly estimate the degree of liver fibrosis through noninvasive evaluation of liver perfusion imaging [20]. A number of studies have shown that liver CT perfusion imaging can reflect changes in blood perfusion in liver fibrosis and early cirrhosis, and the changed perfusion parameters are related to the stage of liver fibrosis, which is of great value for the early diagnosis and treatment of liver fibrosis [21]. Compared with methods using manual feature extraction, deep learning technology can automatically extract regions of interest and features of target images without manual specification and can significantly improve model performance with the help of massive data [22]. The past 2-3 years have seen a dramatic increase in the number of papers applying deep learning techniques to ultrasound disease classification. At the same time, fusing hand-designed features with features computed by deep learning can further improve the performance of the model [23, 24].

RETRACTED

## 3. Methods

### 3.1. Deep Learning

Deep learning is a kind of machine learning, which is an advanced technical means. It completes practical tasks by simulating the connection mode of human nerves. It generally includes several connection layers, and each connection layer is mathematically related to each other. This method is usually based on a large amount of data. By continuously nonlinearizing the data, it establishes abstract high-level features to fit a more accurate model, which is also called hierarchical learning and deep network learning. The perceptron is also the neuron of the model. One neuron corresponds to one output, but the real scene is more complicated. People combine multiple perceptrons to have a perceptron model with multiple outputs. However, the single-layer perceptron model can only be applied to the case where the data are linearly separable, and the data processing in the actual task is linearly inseparable, so the single-layer perceptron model greatly limits its application. From this, researchers began to build a multilayer perceptron model. With each additional model layer, it gets increasingly harder to fit the model. The multilayer perceptron model may now be trained more quickly, thanks to the invention of the backpropagation technique. The ANN was born at this time, which consists of an input layer, an output layer, and several hidden layers. The basic structure of the ANN is shown in Figure 1. The input layer receives incoming data and is made up of neurons that pass the received data to other layers. The number of elements in the input layer should be equal to the number of variables in the dataset, that is, the number of attributes in the dataset. The hidden layer is between the input layer and the output layer, which contains a large number of neurons. As the network continues to train, the weights are updated and the prediction ability is stronger. The output layer integrates the predicted features, which is mainly different from the model type. If the model is a classification network, the output will have multiple values according to the task. If the model is a regression network, the output will have one value according to the task. The weight of a neuron refers to the strength of the connection between two neurons, and the weight is usually initialized to a small value, such as a normally distributed value between −1 and 1.

Deep learning is a learning method that uses deep ANN to solve practical tasks. Compared with shallow network models, it has a layered structure and can use multiple layers of nonlinear changes to abstract features. However, at the same time, its training difficulty is also greatly improved. In the process of deep learning network model training, there are often situations such as overfitting or underfitting. The liver fibrosis degree assessment task in this paper adopts a modeling method based on DNN. Through a large number of nonlinear transformations in the modeling process, an abstract feature map can finally be obtained, that is, the features learned by the network; in the training process, various methods are used to avoid overfitting and underfitting.

### 3.2. Basic Structure of the Convolutional Neural Network

CNN is a common structure in deep learning framework, and its model is the most widely used in deep learning. At the same time, it has a very prominent performance in classification and recognition tasks, so this paper also uses the CNN model combined with the theory of transfer learning to complete the classification and recognition of liver fibrosis. It gives an effect of learning, or the influence of the experience of learning on the completion of other activities. For liver fibrosis images, the input layer of the CNN is passed into the network, the surface damage data features are extracted through one or more layers of convolution pooling and other operations, and the extracted features are then entered into one or more full connection layers. Finally, the damage category label is output through the output layer.

RETRACTED

#### 3.2.1. Convolutional Layer

In a CNN structure, there are usually multiple convolutional layers. The low-level convolutional layer usually obtains the overall information of the image, such as edges and lines, but as the number of convolutional layers increases, more complex and more advanced features can be extracted through continuous iteration. The operation of extracting features from the input image in the convolution layer is called the convolution operation. The relationship between the input and output of the convolution operation is expressed as

(1) $$\begin{array}{c} Y=\frac{1-B+2P}{S}. \end{array}$$

It can be seen from the formula that the output feature map size *Y* is related to the convolution kernel size *B*, the convolution kernel single moving step *S*, the input image size, and whether it is filled.

The above formula is used for a 5*∗*5 image. When using a 3*∗*3 convolution kernel for convolution operation, assuming that the step size of a single movement of the convolution kernel is set to 1, the calculation formula of the feature map size after output convolution is

(2) $$\begin{array}{c} \left\{\begin{array}{c} P=\text{valid}⟶Y=\frac{5-3}{1}+1=3,\\ P=\text{same}⟶Y=\frac{5-3+2}{1}+1=5. \end{array}\right. \end{array}$$

Through the analysis, it can be seen that different choices of filling methods can keep the input image size unchanged or reduce the input image size. For CNNs, the convolutional layer usually adopts *P*=same filling method to maintain the image size. The change of image size is achieved through the pooling layer. It can be seen from the analysis that the stride and the size of the convolution kernel together determine the size of the feature map. The computing speed of the network is determined by the sparse connection and weight sharing between the convolution kernels. Sparse connections are relative to ANNs. In the ANN, each neuron in the current layer is connected to all the neurons in the front and back layers. The drawback is that each link has a weight that must be memorized and stored. Increasing the depth of the network model increases the difficulty of training and converging the network, as well as the amount of memory required to execute the task. In CNN, each neuron simply saves weights in its own structure to address the ANN problem. For example, a convolution kernel of size 3*∗*3 only has to store its own 9 weights; hence, the number of connections between each neuron and the preceding layer is solely linked to its own size. The term “sparse connection” refers to the fact that the convolution kernel has less connections than a fully linked system. For the same convolution kernel, the weights utilized in the convolution operation will be the same in each round of training and the internal weights will only be modified after one iteration has been finished. For a convolution kernel, the weights of each convolution remain the same over each iteration. This is known as weight sharing.

RETRACTED

#### 3.2.2. Pooling Operation

In theory, all feature maps extracted by convolution can be used as the input of the network model, but the result of this is that the increase in the amount of parameters leads to an increase in the amount of calculation, so in the convolution operation when done, a pooling operation is required. By setting the step size and window size, the network further reduces the size of the network and the amount of parameters without changing the number of channels and network weights, so as to divide the entire data through pooling and solve several convolutions. When the layer performs feature extraction, a large amount of computation and parameters are generated, thereby reducing the dimension of the image. The addition of pooling reduces the overfitting of the network to a certain extent and increases the image processing speed, thereby improving the performance of the network model. Commonly used pooling methods are max pooling and average pooling. Among the two pooling methods, max pooling is the most commonly used pooling method. In practical applications, in order to further alleviate overfitting, some pooling layers also use overlapping pooling, which means that the pooling windows are allowed to overlap to form overlapping average pooling and overlapping maximum pooling, which effectively reduces the error rate.

#### 3.2.3. Fully Connected Layer

To put it simply, the full-connected layer uses the fundamental matrix operation to get its result: a one-dimensional vector. It is used to categorize and identify characteristics of a subject. Because of its completely linked function, it frequently has to keep a large number of parameters and uses a large amount of storage space. The convolutional layer can be used instead of the fully connected layer to retain the image's spatial structure while reducing memory usage due to the benefits of the convolutional layer.

RETRACTED

#### 3.2.4. Activation Function

For complex data such as images and audio, the neural network must have the ability to solve nonlinear tasks in order to extract and learn complex features from these data and introduce activation functions to add nonlinear characteristics to the network. Let the model have the effect of fitting the data well. Commonly used activation functions are sigmoid, Tan*h*, and ReLU. The sigmoid function expression is

(3) $$\begin{array}{c} f\left(x\right)=\frac{1}{1+e^{-x}}. \end{array}$$

The sigmoid function nonlinearly maps the input continuous real numbers between 0 and 1. When the sigmoid function is infinitely close to 0 or 1, the function will be saturated, that is, the gradient will disappear, resulting in the inability to calculate the weight, the parameters cannot be updated, and the querying new data cause neural network training to fail. Therefore, the sigmoid function is not used in the probability output of the final CNN.

Tan*h* function is also called hyperbolic tangent function, and its function expression is

(4) $$\begin{array}{c} f\left(x\right)=\frac{e^{x}-e^{-x}}{e^{x}+e^{-x}}. \end{array}$$

The emergence of the hyperbolic tangent function, centered at 0, solves the problem that the output value of the sigmoid function is always greater than 0, but the gradient function still has a saturation phenomenon, that is, the problem of gradient disappearance still exists, when the input value of the function is greater than the fixed value or when it is less than the fixed value, the output value of the function will be fixed at about 1 and −1, which will lead to a small derivative value of the function. At the same time, when the network parameters are updated, according to the chain derivation rule of the derivative, with the network layer increases, the gradient vanishing phenomenon still exists.

The functional expression of the ReLU function is

(5) $$\begin{array}{c} f\left(x\right)=\left\{\begin{array}{c} x,\;x\geq 0,\\ 0,\;x<0. \end{array}\right. \end{array}$$

When the input of the ReLU function is negative, the corresponding function value of the function is 0. When the input value is not negative, the function is a zero-crossing point and a positive proportional function with a slope of 1. Because the ReLU function has a faster convergence speed and with the input when the value increases, the gradient value remains unchanged and the problem of gradient saturation will not occur. Therefore, in most neural networks, ReLU is usually selected as the activation function. However, the problem with the ReLU function is that when the input value is negative, the corresponding function value is always 0. At this time, the gradient saturation will occur and the neurons in the network cannot be activated. However, this problem can be circumvented by setting the learning rate parameter.

RETRACTED

### 3.3. Training of the Network Model

#### 3.3.1. Dropout Strategy

In the classification and recognition network model of liver fibrosis degree, the phenomenon of overfitting is manifested in that the deviation of accuracy between the training set and the test set of liver fibrosis images is too large, so that the network model can hardly be used. The proposal of network sparsification effectively prevents the overfitting phenomenon in the training process. During training, some input nodes or output nodes are randomly disabled. Dropout can be regarded as adding an auxiliary layer with uncertainty to the network, which can reduce the training parameters of the network and improve the generalization ability of the model.

#### 3.3.2. Cross-Entropy Damage Function

The output layer is used for image classification and recognition, and the input images can be classified into corresponding categories in the form of probability. The loss function, also known as the cost function, is used to evaluate the error between the true value of the model and the output value. As the loss value decreases, the stability of the model gradually increases. In this experiment of classifying and identifying the degree of liver fibrosis, the softmax cross-entropy loss function was used to calculate the error. The loss for each batch is

(6) $$\begin{array}{c} J\left(x,\hat{y}\right)=-\frac{1}{m}\sum_{j=1}^{m}\sum_{i=1}^{n}\left[y_{ji}log{\hat{y}}_{ji}+\left(1-y_{ji}\right)\text{log}\left(1-{\hat{y}}_{ji}\right)\right], \end{array}$$

where *m* is the total number of samples and *n* is the number of label categories. If only one iteration of the network model is performed, the loss values obtained by all batches are connected to obtain the loss curve in the training process.

#### 3.3.3. Parameter Optimization Method

The process of network training is the process of updating the weights of the network iteratively, which is also the process of parameter optimization. From the previous section, we know that the network performance is evaluated by the loss function. The better the network performance, the lower the loss value, and the reduction of the loss value is the result of the continuous optimization of the network. Commonly used network optimization methods include mini-batch gradient descent method, momentum technology, and adaptive time estimation method. The mini-batch gradient method solves the frequent update and fluctuation of traditional gradient descent algorithm, resulting in large fluctuations in loss function and network instability and convergence. However, the learning rate of mini-batch gradient descent is fixed, and the same learning rate makes it difficult to converge when the training sample data are sparse. The same momentum technique also faces the problem of nonconvergence of the model caused by the fixed learning rate. The adaptive time estimation method can adjust the learning rate without human participation in the network training process. This method of automatic learning rate adjustment can not only shorten the iteration time required for network training but also improve the learning effect. It can prevent the learning rate from disappearing and reduce the fluctuation range of the loss function. Obviously, compared with other algorithms, Adam is more suitable as a parameter optimization method for liver fibrosis classification and identification experiments.

RETRACTED

#### 3.3.4. Batch Normalization Algorithm

As the depth of the network model built by deep learning increases, the training process of the model becomes more and more complicated and the convergence rate of the network model decreases. Therefore, the batch normalization (BN) algorithm is introduced. For a complex network model, some of the neurons in the hidden layer can also be regarded as input, so the activation value of each hidden layer neuron in the deep neural network can be preprocessed by whitening.

In order to select the optimal network model for experiments, this paper selects four classic models for experimental comparison, including the AlexNet model, the VGGNet-16 model, the VGGNet-19 model, and the GoogleNet model.

### 3.4. Feature Extraction Based on RTE Images

We extracted 11 image features to quantify RTE images, directly obtaining each elastography parameter. The ranges of 11 parameters reflecting liver fibrosis in real-time elastography are shown in Table 1. In addition, we also considered the patient's age and gender as characteristics. Therefore, for each sample, we collected a total of 13 features.

As can be seen from Table 1, the value range of each parameter is different and cannot be directly used to train the neural network model. Therefore, we first normalized the data. For continuous-valued scalars, we normalize them so that each parameter value is in the range [0, 1]. For example, the age of the patient is usually between 0 and 100 years. If the patient is 55 years old, the standard value should be 0.55; the standardization formula is

(7) $$\begin{array}{c} {\bar{x}}_{i}=\frac{x_{i}-x_{\min}}{x_{\max}-x_{\min}}, \end{array}$$

where *x*_*i*_ refers to the value of the input variable, *x*_min_ is the minimum value within the data range, and *x*_max_ is the maximum value within the data range. In addition, for binary variables, 0 and 1 are used to represent features, for example, gender is 1 for female and 0 for male.

RETRACTED

## 4. Experiment and Analysis

### 4.1. Data Sources and Evaluation Indicators

The research subjects were from a multicenter real-time elastography project of hepatitis B fibrosis. A total of 780 patients with chronic hepatitis *B* and cirrhosis participated in this study. The study protocol was approved by the relevant institutional independent ethics committee, the purpose of the study was explained to the patients, and written informed consent was obtained. The inclusion criteria of patients were as follows: (1) they had received histopathological examination of the liver; (2) they had a history of hepatitis *B* or HBsAg positive for more than 6 months and were still HBsAg positive; (3) they had undergone an ultrasound examination. The exclusion criteria were as follows: other types of hepatitis other than viral hepatitis B, metabolic diseases, fatty liver, and drug-induced and alcoholic liver injury. Ultimately, a total of 640 samples were selected for analysis. The study subjects included 480 male and 260 female patients, ranging in age from 22 to 70 years.

According to the classification and identification of the degree of liver fibrosis in this subject, the accuracy of the evaluation index is selected for evaluation, and the formula is

(8) $$\begin{array}{c} \text{Acc}=\frac{\text{number of correctly predicted samples}}{\text{total number of samples}}. \end{array}$$

### 4.2. Best Fit Model Selection Experiment

In order to obtain the most suitable network model, four network model structure schemes were selected in this experiment, namely, AlexNet, VGG-16, VGG-19, and GoogLeNet. By comparing and analyzing the recognition accuracy values of different network models on the test set, the optimal network model structure is selected.  Table 2 shows the recognition results of different network models. From the table, we can see that the recognition accuracy of the GoogLeNet model is better than other models, so the optimal network model selected in this paper is GoogLeNet.

### 4.3. Optimal Model Optimization Experiment

Through the experimental analysis of the optimal model selection, it can be seen that GoogLeNet is the optimal model, but different iterations, batches, and learning rates can lead to changes in the output of the model. In order to verify how many training batches, how many learning rates, and how many network iterations, the GoogLeNet recognition effect is the best and the performance of the network model is verified by controlling variables, so as to select the optimal liver fibrosis degree recognition model.

RETRACTED

#### 4.3.1. Batch Size

In order to verify the influence of different parameters on the classification and identification of wind turbine blade surface damage and then select the optimal GoogLeNet network model parameters, we first conduct batch size experiments. Ideally, the batch size of the network model should be the iterative experiment using the entire training set. However, if the batch size is too large, it will not only affect the network performance, but also increase the computer burden. In this experiment, 16, 32, and 64 were selected as the batch size of the experiment, and the test results were analyzed.  Figure 2 shows the model test results for different batch sizes.

Through the analysis of Figure 2, it can be seen that the introduction of large batches will reduce the performance of the network and the accuracy of 32 batches is higher than that of other batches. Therefore, batch size 32 is selected as the parameter in this experiment.

#### 4.3.2. Learning Rate Setting

In order to explore the influence of different learning rates on the model recognition results, three different learning rates were set, respectively, and the accuracy of the test set under different learning rates was compared, as shown in Figure 3.

Similarly, through the analysis of Figure 3, it is found that the recognition result of 0.001 learning rate is the lowest, which cannot meet the experimental requirements. The accuracy rate of 0.0005 is the highest, so the learning rate of 0.0005 is finally selected as the parameter of the model.

#### 4.3.3. The Number of Iterations Experiment

In order to further optimize the model, we collected the accuracy and loss during the running of the model, that is, the accuracy and loss of the training set and validation set, as shown in Figures 4 and 5.

From Figure 4, it can be seen that, with the increase of the number of iterations, the accuracy of the network is constantly improving and the loss is also decreasing, but the curve does not change significantly after 8 iterations. 8, 9, and 10 were selected as the number of iterations, and the most suitable parameters for the model were selected by analyzing the accuracy of the test set under different iterations.  Figure 6 shows the model test results for three iterations. It can be clearly seen that when the iteration is 10, the recognition effect of the network model is the best.

RETRACTED

## 5. Conclusion

Liver fibrosis is a pathological process of abnormal connective tissue proliferation in the liver, usually caused by various pathogenic factors. Liver fibrosis will occur in the process of liver repair and healing of any liver injury, but if the injury cannot be removed in time, the development of liver fibrosis to a later severe stage will lead to liver cirrhosis, which in turn leads to serious complications such as liver cancer. At present, the diagnosis of liver diseases mainly includes liver biopsy, serum examination, and imaging examination. MRI has advantages in observing and evaluating superficial organs, cartilage, and other tissues and has multiplanar imaging capabilities, but it is expensive and cannot be dynamically checked in real time; compared with CT, it has insufficient spatial resolution and radiation damage, and MRI cannot perform real-time dynamic examination. Ultrasound imaging technology has the advantages of nondestructive, real-time, convenient, and no ionizing radiation and is suitable for clinical screening and follow-up, especially for the diagnosis of liver fibrosis and early cirrhosis, and its advantages are obvious. For the analysis of medical images, the main method is manual interpretation, which depends on the subjective experience and knowledge level of doctors, which is prone to subjective misjudgment and low efficiency. In this context, this paper extracts the characteristic parameters of liver fibrosis ultrasound images and then uses neural network to evaluate the degree of liver fibrosis and completes the following work: (1) it introduces the research background, research significance, research status at home and abroad, and the influence of the development of medical imaging on the diagnosis of liver fibrosis; (2) the related technologies of deep learning and deep convolutional network are introduced, and the indicators of liver fibrosis degree assessment are constructed by using ultrasonic image extraction features; (3) using the collected liver fibrosis dataset to conduct model evaluation experiments, four classic CNN models are selected to compare and analyze the recognition rate. The experiments show that the GoogLeNet model has the best classification and recognition effect.

## Figures and Tables

**Figure 1:** Topological structure of artificial neural network.

**Figure 2:** Comparison of model accuracy under different batch sizes.

**Figure 3:** Comparison of model accuracy under different learning rates.

RETRACTED

**Figure 4:** Training set and validation set accuracy curve.

**Figure 5:** Training set and validation set loss curve.

**Figure 6:** The accuracy of the model under different iterations.

**Table 1:** Liver fibrosis ultrasound real-time tissue elastography parameter index.

Attributes	Attribute value range	Label
Strain mean	53.28–140.35	*X*1
Standard deviation	28.45–74.75	*X*2
Blue field percentage	0.72–61.87	*X*3
Complexity	9.16–58.89	*X*4
Consistency	0–0.05	*X*5
Contrast	64.20–348.95	*X*6
Correlation	0.95–0.99	*X*7
Equality	3.18–4.05	*X*8
Clutter	0.06–0.25	*X*9
Skewness	0.15–1.22	*X*10
Kurtosis	1.96–4.13	*X*11

**Table 2:** Damage identification results of different network models.

Network structure	Acc
AlexNet	0.3895
VGG-16	0.6728
VGG-19	0.8676
GoogLeNet	0.9529

## Data Availability

The datasets used during the current study are available from the corresponding author on reasonable request.
